The article "E-Commerce Information System Management Based on Data Mining and Neural Network Algorithms" was published in 2022. Journal: Comput Intell Neurosci.

# E-Commerce Information System Management Based on Data Mining and Neural Network Algorithms

**DOI:** 10.1155/2022/1499801

**Published:** 2022-04-11

**Authors:** Qing Zhang, Abdul Rashid Abdullah, Choo Wei Chong, Mass Hareeza Ali

**Affiliations:** ^1^School of Business and Economics, University Putra Malaysia, 43400 Seri Kembangan, Malaysia; ^2^Laboratory of Computational Statistics and Operations Research, Institute for Mathematical Research, Universiti Putra Malaysia, 43400 UPM Serdang, Selangor, Malaysia

## Abstract

The rapid development of artificial intelligence technology has led to rapid development in various fields. It has many hidden related customer behavior information and future development trends in the e-commerce information system. The data mining technology can dig out useful information and promote the development of e-commerce. This research analyzes the significance and advantages of data mining technology in the application of e-commerce management systems and analyzes the related technologies of data mining and future trend prediction. This research has taken the advantages of clustering and naive Bayesian methods in data mining to classify product information and purchase preferences and other information and mine the associated data. Then, the nonlinear data processing advantages of neural networks are used to predict future purchasing power. The results show that data mining technology and neural networks have high accuracy in predicting future consumer purchasing power information. The correlation coefficient between real consumption data and predicted consumption data reached 0.9785, and the maximum relative average error was only 2.32%. It fully shows that data mining technology can obtain some unrecognizable related information and future consumption trends in e-commerce systems, and neural networks can also predict future consumption power and consumption patterns well.

## 1. Introduction

In recent years, with the rapid development of high-performance computers, the Internet, and data mining, artificial intelligence technologies such as machine learning strategies have been widely used in human life activities [1]. Similarly, the digital and intelligent transformation of e-commerce management has become the focus of attention in the field of practice and academia, and many entities and companies have made great progress in intelligent e-commerce [2]. Data mining technology can give full play to its own algorithmic advantages and can extract the inherent connection time and space information implicit in the data through algorithms such as clustering and Bessell [3]. The data information of the e-commerce management system is a typical time and space characteristic relationship, and this technology can be applied in the e-commerce system.

In the modern era of big data and electronic information, there is a wide range of highly relevant information in all walks of life. This information and relevance are difficult to find by man, but data mining technology can make good use of this information [4]. Efficiently identifying useful information from the complex and disorderly original data and assisting the e-commerce field in making accurate decisions, realizing the intelligent of e-commerce management systems, will be the general trend in the contemporary e-commerce field. Accurately classifying and summarizing these data and making the development direction of e-commerce management by many data are the primary problems faced by enterprise managers [5]. At the same time, the data and information from inside and outside the enterprise are changing rapidly [6]. The traditional business analysis work can no longer meet the enterprise's demand for information updates. The intelligent e-commerce management model is extremely necessary for the enterprise [7]. Now human beings have made great use of e-commerce business, such as shopping, medical treatment, and office, but these data have not been fully excavated. It makes sense to fully explore the relevance and guide future trends [8].

At this stage, some related research work has been done on big data mining and neural network in the e-commerce management system. Zu et al. [9] used the matrix theory method to study the correlation between customer types and shopping type, which uses mathematical statistics to classify and summarize information such as consumers' daily consumption patterns and brand preferences. The conclusion shows that this method can mine effective and accurate information from a large amount of information between customers and shopping and can help e-commerce companies formulate reasonable and efficient logistics management plans. Through improved IPA model, support vector machine, and Bayesian machine learning algorithms, Luo et al. [10] proposed an online e-commerce management data mining and decision management model that integrates data collection and cleaning, data mining and analysis, and strategy formation and considers consumption. The influence of consumer psychology and other factors on shopping decision-making. Qu et al. [11] applied the advantages of edge computing methods to the evaluation framework of the e-commerce supply chain. At the same time, this model can establish a fuzzy neural network based on the supply chain. The predicted value of the pricing plan is in good agreement with the planned value, which further illustrates the accuracy and feasibility of this method in e-commerce. Lai and Cai [12] used FPGA analysis technology and a large data mining method to establish a China-Japanese cross-border e-commerce management model by the consumer's preference for the work and the characteristics of the work itself. Ghavamipoor et al. [13] proposed a sensitive customer behavior model QoS-CBMG for the service quality of e-commerce platforms, which is used to improve e-commerce customer satisfaction and increase profits. Luk et al. [14] fully excavated potential customer population and behavioral information and established an intelligent customer identification model to formulate the relationship between customers and needs in the shortest possible time. Qi et al. [15] used the classic analysis model KANO to mine online e-commerce product information to get the future trend of product information. Vanderveld et al. [16] used the random forest method to establish a customer lifetime value system based on the value relationship between products and customers and established a customer value system based on purchasing behavior. The system has been deployed to predict the value of hundreds of millions of users every day. This is a successful e-commerce management model. Mach-Krol and Hadasik [17] used advanced big data analysis BDA theoretical methods and traditional system search methods to study the role of big data mining in understanding customer behavior. The results of the study showed that customer behavior has a strong correlation with the time dimension. From the above literature review, it can be seen that most of the studies are mainly aimed at the classification of data in the field of e-commerce [18–20]. They mainly use decision trees and support vector machines, but they do not further predict the data in the field of e-commerce. In this article, based on the characteristics of the collected customer behavior information, the clustering method is used to classify, and the classification results are predicted, which truly realizes the intelligent process of e-commerce information.

With the rapid development of big data technology and e-commerce technology in various industries, many related data that can be mined and utilized have emerged [21]. At the same time, the rapid development of computer technology and hardware equipment has also made it possible for the application of data mining technology and deep learning technology in e-commerce management systems, which is very convenient and efficient for people. Big data collection technology has also been greatly improved [22]. RFM method can describe the value of customers by understanding the customers who have purchased on the website or the degree of customer interest in their products and by analyzing customer behaviors to describe the value of customers, which can be distinguished according to time, frequency, amount, etc., and then it can dig out the characteristics of their behaviors information and can be actively recommended through e-commerce recommendation systems [23]. Due to the rapid development of science and technology, injecting intelligent e-commerce management mode will surely become a historical development trend and an inevitable product of strong market demand [24]. Neural networks have great advantages in predicting future trends, and there is more potential information in e-commerce management, which is beneficial to e-commerce management [25].

This article is mainly composed of five chapters. The detailed introduction is as follows: the first part introduces the development of the e-commerce management system and the research of data mining technology and neural network in e-commerce related aspects. The second part introduces the significance and advantages of data mining and neural network technology in the application of e-commerce management systems and the way to obtain data sets. The third part explains the methods of data mining such as clustering, the theory of neural network technology, and the method of data normalization. The fourth chapter focuses on the analysis of neural network technology to predict future consumer purchasing power and purchasing trends and conducts an intuitive analysis through statistical parameters. The fifth section is the summary part of the article.

## 2. The Significance of E-Commerce Information System and Data Mining

### 2.1. The Significance of Data Mining for E-Commerce Information System

For the e-commerce system using data mining technology, it can fully extract the relationship between various features and at the same time can extract data that cannot be obtained by human work [26]. For example, for e-commerce managers, they can obtain customers' purchase amount, purchase quantity, purchase frequency, and other information through their own website system, but it is difficult for humans to directly establish some connections with these scattered variables, which makes it difficult to find the connections and relevance among them [27], which is very unfortunate for e-commerce practitioners. If you can make full use of these data, dig out the links between these data from the data, and guide the future development trend and business model of the enterprise or company, it is a very meaningful thing [19]. It can not only guide e-commerce managers to make more appropriate business strategies [28] but also predict the purchase behavior of future customers in time to improve the competitiveness of their products. At the same time, it can also provide sales staff with more data support and important customer resources, which is also meaningful for sales. In general, it is a meaningful and competitive business for how to use the correlation between big data and guide future development and marketing strategies in the era of big data [29]. For enterprise-type e-commerce, there are different types of data and many customers. These cumbersome data are difficult to count and even more difficult to find the rules. At the same time, for some e-commerce products, their laws may be related to the development of seasons or weather, which is even more impossible to discover by manual statistics [30]. Through the continuous efforts of computer staff, data mining technology and algorithms have been rapidly developed, and a wide variety of clustering or data mining algorithms based on probability prediction have appeared, and these algorithms have different applicability [31]. At the same time, it provides more choices for e-commerce data mining and neural network prediction technology. In order to improve the efficiency of e-commerce practitioners and improve the company's ability to predict future trends, data mining technology is an intuitive and important means [32]. Therefore, in the era of rapid development of big data and unmanned technology, finding the most suitable data mining technology and neural network prediction model suitable for enterprises and customers is a challenging and meaningful work, which can not only be useful for sales staff providing greater welfare space can also bring more benefits and far-reaching development to the enterprise [29]. At the same time, data mining technology has brought many benefits to many large enterprises and more consumers, which is a trend that cannot be ignored [33].

### 2.2. The Preparation of Datasets and Data Cleaning

Both neural networks and data mining methods have strict requirements on datasets, and bad datasets will seriously affect the accuracy of prediction. Although data preprocessing is the basic work of learning, it is also an extremely critical step. The data preparation process can be divided into two processes: data selection and data preprocessing. The purpose of data selection is to determine the associated data for discovery-related tasks, such as customer purchase frequency and purchase value. In the field of e-commerce, operators are more concerned about the profit and loss status of e-commerce. The factors that have a greater correlation with the profit and loss status are mainly the sales of goods, the frequency of purchases by customers, and the number of purchases. Therefore, this article selects customers' purchase frequency, purchase preference, and purchase amount. These datasets reflect the performance of e-commerce more intuitively. The data prediction process generally includes eliminating noise data, calculating missing values, and completing data type conversion. In real life, the integrity of the data set is difficult to guarantee, and some data points may be missing. This requires supplementary work for missing data according to the situation, which has reached the data format required by the machine learning method. The collected data must have similar distributions, and the emergence of extreme values must be avoided, which will lead to excessive prediction errors. The dataset is mainly composed of the customer's consumption amount, consumption frequency, and type of products purchased, which serves as the input layer of the neural network. The value of consumers is the output layer of the neural network. The processing process of the data set in the data mining and neural network prediction process is shown in Figure 1. It can be seen that preprocessing operations such as data cleaning are performed for the collected data, and then the availability and accuracy of the data are explored, and finally the collected data are input through the model.

## 3. Method and Theory

### 3.1. Data Mining

Data mining technology refers to the automatic classification technology that finds more relevant categories from a large amount of collected data. At the same time, the collected data have a big difference in characteristics, which is also the preprocessing data process of data mining [34, 35]. Find the optimal classification process through methods such as clustering, decision tree, and self-defined model hyperparameters. Then, it can be fully utilized to find the connection between the data and can be used as the basic data to predict future customer behavior. Nondependent data is relatively simple, which is commonly referred to as multidimensional data [36]. Dependent data, the so-called dependency, is a relationship between data items that has a certain correlation change. Data mining specifically divides this relationship into implicit dependence and explicit dependence.

The application of data mining technology in e-commerce is very suitable. E-commerce information not only has the correlation between characteristics, such as the relationship between customer purchase product data, consumption amount, and personal consumption frequency or season. At the same time, the field of computer science has provided many open-source algorithm libraries and guiding methods that can be used for e-commerce management data mining strategies. For data from different sources, you can make changes according to different algorithm rules and finally find an algorithm that suits your own data characteristics.

### 3.2. Clustering Theory

Clustering is a commonly used unsupervised learning category in the field of machine learning. It can classify different categories according to the relevance of the data. Clustering is the process of dividing a dataset into different categories according to a certain criterion (such as distance and density). The data between the same category have strong similarity and the difference between different categories is as large as possible. The process of clustering optimization is also a process of continuously approximating the similarity between the same classes and continuously increasing the differences between different classes. According to the different clustering methods, it can be divided into partition clustering methods, density-based clustering methods, hierarchical clustering methods, and so on. In this article, according to the feature relationship between the datasets, the partition clustering method is selected as the method of data mining.  Figure 2 shows the method of K-means, and Figure 3 shows the density-based clustering method. In this study, the method of K-means was used to study e-commerce. Although clustering is a mature classification method, most of the classification problems in the field of e-commerce use support vector machines and decision trees, and there are relatively few studies using clustering methods [34], which may be related to the selected e-commerce dataset. In this article, the clustering method based on the distance method is used to study the application in e-commerce, which is innovative to a certain extent [37, 38].

The training datasets, testing datasets, and predicted value can be described as (1)–(3). To better evaluate the accuracy of the datasets divided by clusters, three distance evaluation indicators are introduced for the analysis. The measurement standard of clustering is generally measured by the distance method, and there are probably three ways of judging distance. *x* is the input dataset, *y* is the output value, and $\hat{y}$ is the predicted value.

(1) $$\begin{array}{c} \text{Train}=\left\{\left(x_{1},y_{1}\right)\left(x_{2},y_{2}\right),\ldots ,\left(x_{n},y_{n}\right),\ldots \left(x_{N},y_{N}\right)\right\}, \end{array}$$

(2) $$\begin{array}{c} \text{Test}=\left\{\left(x_{1},y_{1}\right),\left(x_{2},y_{2}\right),\ldots ,\left(x_{m},y_{m}\right),\ldots \left(x_{M},y_{M}\right)\right\}, \end{array}$$

(3) $$\begin{array}{c} \hat{y}=\left\{{\hat{y}}_{1},{\hat{y}}_{2},\ldots ,{\hat{y}}_{m,}\ldots ,{\hat{y}}_{M}\right\}. \end{array}$$

The distance of the Minkowski method is where *x* is the input vector, *y* is the output vector, and *p* is the number of clustered categories. In this study, *p* = 4 or *p* = 5, which is to verify the impact of the number of categories on the clustering effect so as to select the best classification standard based on customer behavior. *x* is the input dataset and *y* is the real value.

(4) $$\begin{array}{c} d\left(X,Y\right)=\sqrt[{p}]{{\left|x_{1}-y_{1}\right|}^{p}+{\left|x_{2}-y_{2}\right|}^{p}+{\left|x_{3}-y_{3}\right|}^{p}+\ldots +{\left|x_{q}-y_{q}\right|}^{p}}. \end{array}$$

The distance of the Euclidean method is the special case of Minkowski method when *p* = 2. This form is similar to the evaluation index of average error, which is also a commonly used evaluation index.

(5) $$\begin{array}{c} d\left(X,Y\right)=\sqrt{{\left|x_{1}-y_{1}\right|}^{2}+{\left|x_{2}-y_{2}\right|}^{2}+{\left|x_{3}-y_{3}\right|}^{2}+\ldots +{\left|x_{m}-y_{m}\right|}^{2}}. \end{array}$$

The distance of the Manhattan method is the special case of the Minkowski method when *p* = 1.

(6) $$\begin{array}{c} d\left(X,Y\right)=\left|x_{1}-y_{1}\right|+\left|x_{2}-y_{2}\right|+\left|x_{3}-y_{3}\right|+\ldots +\left|x_{n}-y_{n}\right|. \end{array}$$

### 3.3. CNN Neural Networks

The dataset in the field of e-commerce is huge and cumbersome. If a fully connected neural network is used, it will consume a lot of computing resources and computing time, which is unfavorable for practical applications in the field of e-commerce [39–41]. CNN has the advantage of weight sharing, which can greatly reduce the computational complexity, and it can extract important features well. It is also easy to implement on the TensorFlow platform. This article reduces the computational complexity by setting a larger number of filters and a larger learning rate. CNN has obvious advantages in extracting data features and has been widely used in image recognition, target detection, and other fields. It is a relatively mature algorithm. There are many customer characteristics in the e-commerce management system, such as the customer's purchase type and purchase amount, which are vital to the prediction of customer value. The CNN can effectively extract the features, perform nonlinear operations to obtain a certain mapping relationship, and then predict the future purchase behavior. This method is suitable for the feature extraction and prediction process in e-commerce.  Figure 4 shows the process of CNN. The CNN can perform convolution operations according to the number of filters and sliding steps set by the model [42], and it can then perform the model prediction output through the pooling layer and the activation function layer and finally compare it with the real one. At the same time, the gradient is minimized according to the loss function and the backpropagation method, and finally, the optimal weight parameter is found for the customer information of the e-commerce management system to predict the future trend. Once the model is trained, the model's weights, biases, and hyperparameters are determined. In real-world prediction, some data in e-commerce are collected, and the corresponding mapping value can be output directly through this model, which is consistent with the output in the simulation, but in real operation, it is no longer necessary to train this model, which saved a lot of time. CNN has been proven in many fields to have good performance in extracting data features. At the same time, this article uses the TensorFlow platform and Keras for training and testing [37, 43]. The number of filters used in this article is 128, and the learning rate is 0.001. At the same time, the optimization method of gradient descent is used to carry out the backpropagation process. At the same time, the number of layers of CNN used in this article is 5.

The forward propagation and backpropagation processes of the CNN are shown in equations (7)–(12). This is the process of convolutional layer doing convolution operation (as shown in (7)); the ^*∗*^ symbol represents the convolution operation process. This process can be described as follows: first, the convolution kernel *k*_*ij*_^*ζ*^ and the feature *x*_*i*_^*ζ*−1^ perform the convolution operation, then the bias parameter *b*_*j*_^*ζ*^is added, and the excitation value of the activation function is the output parameter of the convolution layer. *x*_*j*_ is the output value and *f* is the mapping function.

(7) $$\begin{array}{c} x_{j}=f\left(\sum_{i\in M_{j}}x_{i}^{\zeta -1}*k_{ij}^{\zeta }+b_{j}^{\zeta }\right). \end{array}$$

This is the residual calculation process of the feature. The function of this function up(*x*) is to reshape the shape of *δ*_*j*_^*ζ*+1^ into the same shape as *δ*_*j*_^*ζ*^ so as to facilitate the convolution operation.

(8) $$\begin{array}{c} \delta_{j}^{\zeta }=\beta_{j}^{\zeta +1}\left(f^{\prime }{\left(u\right)}_{l}^{\zeta }\circ \text{up}\left(\delta_{j}^{\zeta +1}\right)\right). \end{array}$$

The following equation shows the calculation process of the gradient, where *b*_*i*_ is the bias, *δ*_*j*_^*ζ*^ is the weight parameter, *W* is the weight, and *b*_*i*_ is the bias:

(9) $$\begin{array}{c} \frac{\partial W}{\partial b_{j}}=\sum_{u,v}\delta_{j}^{\zeta }uv. \end{array}$$

The following equation shows the derivative of the bias parameter *k*_*ij*_^*ζ*^, which is a parameter in the form of a matrix:

(10) $$\begin{array}{c} \frac{\partial E}{\partial k_{ij}^{\zeta }}=\sum_{u,v}{\left(\delta_{j}^{\zeta }\right)}_{uv}{\left(p_{i}^{\zeta -1}\right)}_{uv}. \end{array}$$

Equation (11) shows the sampling operation process of the pooling layer, where sampling includes maximum pooling and average pooling methods. The function down(*x*_*j*_^*ζ*−1^) is to sum the eigenvalues. Then, it adds a bias to output according to the activation function.

(11) $$\begin{array}{c} x_{j}=f\left(\sum_{u,v}\beta_{j}^{\zeta }\text{down}\left(x_{i}^{\zeta -1}\right)+b_{j}^{\zeta }\right). \end{array}$$

The following equation is the calculation process of the pooling layer to solve the parameters, where *f*′ represents the derivative of the above pooling layer function (11):

(12) $$\begin{array}{c} \delta_{j}^{\zeta }=f^{\prime }\left(u_{j}^{\zeta }\right)\circ \text{conv}2\left(\delta_{j}^{\zeta +1},\text{rot}180\left(k_{j}^{\zeta +1}\right)\right.. \end{array}$$

### 3.4. Data Normalization Processing and Uncertainty Analysis

There are many characteristics in collecting e-commerce customer information, which is disadvantageous for the dataset itself. At the same time, there are obvious differences in the characteristics of the customer purchase amount, type of product purchased, and purchase frequency collected from various channels. This is unfavorable for the operation of neural networks and clustering algorithms. The neural network operation process is to constantly find the weights between the datasets that can represent the best correlation, so the datasets need to be normalized. Normalizing the input data with better distribution characteristics and correlation can speed up the convergence speed and improve the prediction accuracy.

At the same time, when an unknown customer behavior is used as an input layer and predicts future buying behavior trends, there is a lot of uncertainty. In order to avoid the neural network's overconfident prediction process, this article needs to quantitatively evaluate the uncertainty of the prediction process. In the following equation, the variational Bayesian method is used to perform uncertainty analysis, where KL(*q*(*ψ*))‖(*p*(*ψ*) is the process of minimizing the actual posterior distribution *p*(*ψ*) and the variational posterior distribution *q*(*ψ*):

(13) $$\begin{array}{c} \text{VB}=\sum_{l=1}^{L}\int q\left(\psi \right)\ln\;p\left(Y^{N}\right.|X^{n},\left(\psi \right)d\psi -\text{KL}\left(q\left(\psi \right)\left\|\;\right.p\left(\psi \right)\right.. \end{array}$$

## 4. Result Analysis and Discussion

Figure 5 shows the calculation process of customer purchasing behavior clustering. The customer purchase product type, purchase frequency, and purchase amount are used as the basis for classification. As shown in Figure 5, first, customize the number and distance of clustering categories. The clustering algorithm continuously adjusts the gap and related distances between different categories and finally finds the optimal cluster class way. Figures 6 and 7, respectively, show the clustering results of customer purchasing behavior under the conditions of nonuncertainty analysis and uncertainty analysis conditions. It can be clearly seen that customer behavior information is better clustered under uncertain conditions. It can be seen from Figure 6 that the difference between the four different customer behaviors is small, which shows that the clustering effect has not reached the effect of the large difference between the different categories. However, the clustering effect produced by this method performs better in the same category. Under the condition of uncertain analysis, the neural grid is no longer overconfidently predicting unknown values. It can be seen from Figure 7 that the clustering effect on customer behavior is better than that in Figure 6. This clustering method not only clusters closely related categories together but also makes the difference between different categories as large as possible. This is a better clustering method. Through the comparison of Figures 7 and 8, it can be found that the optimized algorithm has better classification performance, and it can clearly segment the consumption value in e-commerce with high correlation, rather than the situation of mutual intersection in Figure 7.

Figure 8 shows the iterative process of the loss function of the training and test sets. In order to more intuitively verify the feasibility and accuracy of the neural network in predicting the e-commerce management system, Figures 9 and 10, respectively, show the heatmap of the predicted value and the error heatmap for different times and different customer groups. It can be seen from Figure 9 that, in general, the data after the clustering process are predicted by the CNN, and the customer value prediction is relatively accurate. Moreover, it not only predicts the value of individual customers's purchase behavior in different months but also predicts the differences between different groups of customers. At the same time, this trend of changes is also predicted well. The above description can show that this neural network model is in the e-commerce management system predicts the trend problem with very good feasibility.  Figure 10 shows the error thermal cloud diagram, where the error of the prediction result of customer value is relatively small, and they are all within the acceptable range. In general, the forecast errors from March to July are relatively large, which may be due to the complexity and variability of summer customer shopping behavior. This conclusion is also consistent with the characteristics of actual shopping behavior, which is a behavior with seasonal characteristics. In order to improve the accuracy of prediction, the neural network model can be improved with more sample characteristics in summer when the seasonal behavior is strong; it is to learn more complex behavior characteristics.  Figure 11 shows the predicted value and true value of customer value.

In order to further visually show the predictive ability of neural networks in the e-commerce management system, Figures 12 and 13 show the scatter plot of linear correlation coefficients and the error histogram, respectively. The linear correlation coefficient reflects the correlation between the predicted value and the true value. The closer its value is to 1, the better the prediction effect is. It can be clearly seen from Figure 10 that there is a strong correlation between the predicted value of customer behavior value and the true value, and its value has reached 0.9785, which is already a good correlation value. At the same time, the distribution range of the error can also be seen through the linear correlation coefficient graph. As described in Figure 10 above, the predicted value from March to July clearly deviates from the linear straight line, while in other months, it shows a better linear correlation. They are all distributed on both sides of a linear straight line. The error histogram reflects the average value of the error, which can reflect the forecast error in a macroscopic view. It can be seen intuitively from Figure 13 that the errors are within an acceptable range, and the maximum error is only 2.32%. This error value is already a good error in the e-commerce field. At the same time, the change trend between the forecast error and the month can also be clearly seen from the error histogram. The neural network model can not only predict the value of a single group or a single month but also better predict the change trend of customer value over the month. From Figure 12, it can be clearly seen that the linear correlation between the predicted value and the actual value of e-commerce is relatively good, basically exceeding 0.95, which indicates that the predicted value of e-commerce is in good agreement with the actual data. At the same time, these e-commerce data points are evenly distributed on both sides of the linear function, and the distances are relatively close.

## 5. Conclusion of the Research

With the development of information technology and big data, e-commerce technology has developed rapidly. Making full use of the predictive capabilities of data mining technology and neural network technology is beneficial to the e-commerce management system. It has the ability to dig out consumer preferences and purchasing power of products and other information, and it also can predict future trends based on this potential related information, which is very beneficial and meaningful for the development of enterprises and even companies.

Classification and prediction in the field of e-commerce is a tedious task. At present, most of the classification and prediction of e-commerce use related machine learning algorithms such as decision trees and support vector machines, but there is no research on the prediction of classification results. Combined with the characteristics of the collected datasets such as customer purchase frequency, customer purchase amount, and purchase preferences, this article uses distance-based clustering to classify and combines CNN to predict the classification results, which is useful for classification and e-commerce in the field of e-commerce. The prediction has a certain practical application value. In this study, it first uses data mining techniques such as clustering and naive Bayes to classify consumer purchase information to dig out relevant information, then use neural networks to predict consumers purchasing power in the future, and get a good result. Regarding forecast performance, although the two clustering methods both show better clustering results, from the perspective of the relevance of similar categories and the effects of categories with larger differences, the clustering method with uncertainty analysis will reflect a better classification effect. The clustering method selected in this article and the setting of the initial value have a good reference value for developing an e-commerce management system. It can be seen that the effect of clustering four different customer values is very obvious. Similarly, the CNN selected in this article is used to extract and predict the value of customer behavior and also reflects a good predictive ability. It can not only reflect the purchase behavior trends of different months and different customer groups but also reflect the seasonal characteristics of purchase behavior. The linear correlation between the predicted value and the true value of the customer value standard has also reached a high degree of accuracy, and its value has even reached 0.9785. The error of the predicted value is within 5%, which is an acceptable range for the e-commerce management system. In general, this article predicts the value of customers based on customer behaviors. According to the selected clustering method and neural network model, it shows good prediction and classification capabilities, which is also a good reference value for other e-commerce management fields.

## Figures and Tables

**Figure 1:** The processing process of dataset in data mining and neural network prediction.

**Figure 2:** The method of K-means.

**Figure 3:** The method of density.

**Figure 4:** The CNN processing.

**Figure 5:** The calculation process of customer purchasing behavior clustering.

**Figure 6:** The calculation results of customer purchasing behavior clustering.

**Figure 7:** The calculation results of customer purchasing behavior clustering at optimized conditions.

**Figure 8:** Training and testing the loss function.

**Figure 9:** The customer behavior value prediction heatmap in different months.

**Figure 10:** Heatmap of predicted value error in different months and customer groups.

**Figure 11:** Predicted value and true value.

**Figure 12:** The linear correlation coefficient.

**Figure 13:** The histogram of prediction relative average error.

## Data Availability

The data used in this article can be reasonably requested by readers and researchers.
